RETRACTED

# Comparison and Economic Envelope Structure Schemes for Deep Foundation Pit of Subway Stations Based on Fuzzy Logic

**DOI:** 10.1155/2022/1148856

**Published:** 2022-07-31

**Authors:** Puzhen An, Ziming Liu, Baoxin Jia, Quan Zhou, Fanli Meng, Zhixin Wang

**Affiliations:** ^1^School of Civil Engineering, Liaoning Technical University, Fuxin 123000, Liaoning, China; ^2^China Railway 16th Bureau Group Co., Ltd., Beijing 100018, China; ^3^China Railway 22th Bureau Group Co., Ltd., Beijing 100043, China

## Abstract

Since the 1990s, with the continuous advancement of urbanization, the proportion of urban population has gradually increased. There is a serious shortage of land resources, and people's demand for underground space is increasing day by day. The construction of subway stations has developed into an inevitable trend in the future construction engineering industry, and it is also necessary to select the best solution from various solutions. The purpose of this paper is to study how to evaluate and analyze the economy of the deep foundation pit envelope structure of subway stations based on fuzzy logic, so as to choose the optimal and most economical plan. This paper proposes a fuzzy comprehensive evaluation method based on fuzzy logic, which is a reasonable method for the classic evaluation index. The experimental results of this paper show that in 2015 about 8% of people chose to travel by subway. By 2020, 54.5% of people chose to travel by subway, an increase of 46.5% during this period. It can be seen that more and more people are willing to take the subway, and subway transportation is a public transportation mode with large transportation volume. It has obvious public welfare, and it can relieve the urban traffic pressure very well, so the investment in subway construction in various cities is also increasing.

## 1. Introduction

With the high densification of cities and the increase of traffic demand, the development of urban underground engineering and the full utilization of underground space have become the trend of alleviating traffic congestion in major cities in China. The deep foundation pit enclosure project is the foundation of subway station development and the focus of construction. It is very important to discuss the safety of the deep foundation pit enclosure of the subway station, and it is also a necessary condition to ensure the safety of the subway station project. In the construction process of deep foundation pit enclosure, choosing the best solution is undoubtedly a major issue, and it is also one of the important issues for the success of construction.

In recent years, with the large-scale emergence of deep foundation pit enclosure projects, its complexity and technical difficulty are also increasing. This will put forward higher requirements for the design and construction of deep foundation pit enclosure engineering. The enclosure of deep foundation pits is not only required to be safe, reliable, stable, and reasonable but also economical and affordable and also needs to control the impact on the surrounding environment. Therefore, it is very important for the smooth implementation of the project to study and analyze the comparison and selection of the enclosure structure of the deep foundation pit of the subway station.

RETRACTED

The innovation of this paper is as follows: (1) This paper introduces the basic content of fuzzy logic and deep foundation pit enclosure of subway stations and focuses on several types of deep foundation pit enclosures for subway stations. (2) This paper summarizes the importance of the comparison and economic analysis of the deep foundation pit envelope structure of the subway station. Through experiments, it was found that Scheme A is the safest and most economical scheme.

## 2. Related Work

With the increasing speed of population growth in recent years, causing traffic jams, in order to relieve traffic pressure, people began to develop underground transportation. Underground transportation such as subways began to appear in large numbers, but the research on the envelope structure of deep foundation pits in subway stations is not deep enough. YouYou et al. found that in the strata, the deep foundation pit built by the underground transportation hub has two confined aquifers and one aquifer. In order to ensure the safety of foundation pit construction, he conducted experiments on odor pumping for hydraulic conductivity and designed two schemes for construction [1]. Zheng et al.'s analysis of piling behavior has been frequently used in deep foundation pits in subway stations. However, few studies have paid attention to the impact of pile cutting on the building envelope. Taking a deep foundation pit in Xi'an as an example, he established a three-dimensional numerical model. He analyzed the soil pressure in the foundation pit and the stress change of the envelope structure under local stress [2]. Hu was developing in many cities and the construction of subway stations is developing faster and faster. This also made deep foundation pit engineering widely used. Due to the tight land use, there will inevitably be existing buildings or structures around the deep foundation pit. So, he analyzed the influence law of deep foundation pit excavation on the envelope structure and pile foundation through finite-element numerical simulation [3]. Lei and Gong found that the design of the envelope structure of the deep foundation pit of a subway station is a multidisciplinary problem, which may lead to a series of safety problems in the actual construction project. Moreover, the excavation of large-scale deep foundation pits will face many difficulties. In order to improve the deep foundation pit engineering, deformation can be accurately predicted, so to ensure the safety of the construction process, he carried out research and analysis on the traditional MSD theory [4]. Yuan et al. found that water is one of the main risk factors for large excavations. The risk of deep foundation pits increases if water seeps into the formation. He used MIDAS/GTS software to carry out numerical simulation on the example of subway deep foundation pit engineering. The results show that the deeper the water in the deep foundation pit, the greater the danger [5]. Bian et al. found that in the excavation of deep foundation pits in subway stations, if the protective measures are not perfect, the safety of subway tunnels will be seriously threatened. So far, the protective effect obtained by using partition excavation in large deep foundation pits is not clear. He performed 3D numerical analysis and combined the constitutive model of the study to study the protective effect of partition wall excavation [6].

RETRACTED

Since the development of deep foundation pit engineering, the traditional enclosure methods (mainly grading and excavation and simple enclosure) can no longer meet the requirements of modern foundation pit engineering. Especially since the reform and opening up, the country has been opened, the economy has developed rapidly, the population has grown, and the urban population has been densely populated. Large-scale high-rise and superconventional buildings and underground works continue to emerge. Therefore, the traditional deep foundation pit enclosure structure scheme can no longer meet the needs of today's social development. Especially around the subway, it should select the optimal plan and the most economical plan for the deep foundation pit enclosure structure plan, so as to meet people's needs. Scholars have a certain understanding of deep foundation pits. However, they did not select the optimal solution, nor did they take into account the economics of the deep foundation pit envelope. Therefore, on this basis, based on fuzzy logic, this paper compares and selects the scheme of the deep foundation pit envelope of the subway station as well as analyzes the economy.

## 3. Fuzzy Comprehensive Evaluation Method Based on Fuzzy Logic

### 3.1. Development Trend of Deep Foundation Pit Enclosure

The foundation pit enclosure project is generally developing in a deeper and larger scale, and the surrounding environment of the foundation pit enclosure is becoming more and more complex. The foundation pit enclosure forms and research methods are in full swing, and the requirements for the foundation pit enclosure structure are getting higher and higher [7]. The main function of the deep foundation pit supporting structure is to retain soil. It enables the foundation pit to be carried out safely and smoothly in the whole process of excavation and foundation construction and ensures no harm to adjacent buildings, public facilities, and surrounding environment. Therefore, the development trend of foundation pit engineering is summarized as follows.

RETRACTED

In the past, the design of foundation pit enclosure works as long as it can meet the requirements of strength control and rarely considers the impact on the surrounding environment. However, in the practice of foundation pit engineering, in many areas with soft soil, ground buildings and underground pipelines are often damaged. However, the building envelope showed no signs of damage. Therefore, the envelope structure should not only meet the strength requirements of the envelope structure but also meet the deformation requirements [8]. The schematic diagram of the deep foundation pit enclosure is shown in Figure 1:

As shown in Figure 1, now the foundation pit designers design and calculate according to the traditional assumed working conditions, which do not closely combine the foundation pit design and construction. The lack of communication and communication between designers and the on-site construction team will cause inconsistencies between the calculation of many projects and the actual project, resulting in unnecessary losses [9].

### 3.2. Common Types of Deep Foundation Pit Enclosure Structures in Subway Stations

With the rapid development of economy and technology, the global construction industry has also achieved rapid development and progress and has made great achievements [10, 11]. Especially the underground building structure, in just a few decades, the development of the subway is getting faster and faster. In the face of the rapid increase of urban population, the construction of underground buildings can not only effectively use space and reduce building footprint but also reduce urban construction investment [12].

#### 3.2.1. Grading and Excavation

Generally speaking, when digging a foundation pit, the foundation soil quality is good, the excavation depth is shallow, the construction site has enough land preparation, and a moderate gradient suitable for the foundation pit project is selected. Grading and excavation are sometimes combined with other enclosure forms to form a simple enclosure that is often used, as shown in Figure 2.

RETRACTED

As shown in Figure 2, grading and excavation are one of the ancient foundation pit support forms. The safety level of the sidewall is suitable for three foundation pits, which has the advantages of low cost and simple structure. The disadvantage is the large amount of excavation and backfilling [13].

#### 3.2.2. Soil Nail Wall Enclosure Structure

Soil nailing is an in situ soil reinforcement technique. The slope of the foundation pit is reinforced with soil nails made of steel bars. If the soil layer of the foundation pit is sand and silt soil, it is not suitable to use the support shape of the soil nail wall. Soil nail enclosures are generally used to support a depth of not more than 18 meters, as shown in Figure 3.

As shown in Figure 3, the soil nailing wall enclosure structure has the characteristics of material saving, low cost, and short construction period. During the construction process, it drives soil nails of certain strength into the soil on site and injects cement slurry or grout. The nails and the slope of the foundation pit form a gravity retaining wall that reinforces the soil, supporting the water and soil pressures generated during the excavation of the foundation pit [14].

#### 3.2.3. Internal Support Envelope Structure

The internal support system is suitable for wall-type enclosures and pile-type enclosures composed of reinforced concrete materials. The inner support structure refers to the internal support system to bear the Earth pressure from the retaining piles or walls. The schematic diagram of the inner support envelope is shown in Figure 4.

As shown in Figure 4, the internal support structure mainly has the following advantages: it is easy to manage the construction quality, the safety and stability are relatively high, the performance of raw materials can be fully utilized, and the foundation can meet the economical and reasonable requirements and be suitable for various conditions [15]. The inner support envelope structure is not limited to the depth of the foundation pit and can be applied to the engineering of the foundation pit with a higher safety level.

### 3.3. Fuzzy Comprehensive Evaluation Method

Fuzzy comprehensive evaluation method is a comprehensive evaluation method based on fuzzy mathematics. The comprehensive evaluation method transforms qualitative evaluation into quantitative evaluation according to the membership degree theory of fuzzy mathematics. The algorithm has the characteristics of clear results and strong systematicness. Through continuous and careful investigation and practice, it has been found that some objective factors are characterized by uncertainty, which will affect the quality of evaluation. Therefore, it introduces fuzzy set theory to form fuzzy evaluation to solve this problem. Since there are many factors affecting the scheme of the deep foundation pit envelope of the subway station, it has the characteristics of ambiguity, so this paper chooses fuzzy logic to evaluate the scheme [16].

RETRACTED

Fuzzy comprehensive evaluation method is an effective method to comprehensively evaluate and make decisions under the influence of multiple factors, and it can also become fuzzy multivariate decision-making or fuzzy comprehensive decision-making [17]. Through fuzzy operation, it makes a comprehensive evaluation.

The mathematical models of fuzzy comprehensive evaluation include two-level and multilevel models. When the factor is two levels, it is further divided into AA to obtain the factor set of the second level as

(1) $$\begin{array}{c} U_{i}=\left\{U_{i1},U_{i2},U_{ij}...,U_{is}\right\},i=1,2,...,m;j=1,2,...,s. \end{array}$$

The divided set also satisfies

(2) $$\begin{array}{c} \overset{s}{\underset{j=1}{\cup }}U_{ij}=U_{i}. \end{array}$$

When the level of the factor set is above the second level, it can also continue to be divided, and then the set composed of the schemes to be evaluated is given as

(3) $$\begin{array}{c} V=\left\{u_{1},u_{2},...,u_{n}\right\}. \end{array}$$

In the comprehensive evaluation, it should be carried out from the bottom. The three basic elements of the fuzzy comprehensive evaluation model are the factor set, the evaluation set, and the single factor evaluation [18].

Therefore, the fuzzy map f can determine a fuzzy matrix *R* ∈ *μ*_*n*×*m*_, which is called the judgment matrix as

(4) $$\begin{array}{c} R=\left[r_{ij}\right]=\left[\begin{array}{cccc} r_{11} & r_{12} & ... & r_{1m}\\ r_{21} & r_{22} & ... & r_{2m}\\ ... & ... & ... & ...\\ r_{n1} & r_{n2} & ... & r_{nm} \end{array}\right]. \end{array}$$

It is composed of fuzzy sets of all single-factor evaluations to represent the affiliation of *r*_*ij*_ and *v*_*ij*_.

### 3.4. Optimal Index System of Deep Foundation Pit Enclosure Scheme

#### 3.4.1. Feasible Enclosure Plan

According to the actual situation of the site, this paper only selects a section of the foundation pit that is relatively open to the proposed foundation pit for analysis. There is wasteland around the foundation pit, and the selected site has a large construction space. Combined with the successful case of deep foundation pit enclosure in a subway station in a certain area, the engineering geological analogy method is used to analyze the foundation pit enclosure in this section. Three different forms can be selected as follows:

  Scheme A: the upper 4.4 m adopts the composite enclosure scheme of 1 : 0.4 grading soil nail wall +15 m slope protection pile +3 prestressed anchor cables. The enclosure technology of this scheme has been widely used in the enclosure of surrounding foundation pits. There is a 2 m thick miscellaneous fill in the upper part that is directly enclosed with piles to the top, and the upper piles bear less force, which will cause a lot of waste, and crown beams are added to the top of the piles. If it is added on the surface, according to a large number of foundation pit enclosure monitoring, it is found that the maximum pile moment is located in the middle and upper parts of the foundation pit. Therefore, the upper part is appropriately grading, the lower part is cast-in-place piles, and the top of the pile is added with a crown beam to make the whole enclosure as a whole. It greatly increases the stability of the enclosure structure, and the amount of earthwork backfill is not large, so that the lower structure has a relatively open space during construction.
  Scheme B: the composite enclosure scheme consists of soil-nailed wall enclosure and prestressed anchor cables. This scheme does not require large-scale piling machinery, the construction process is relatively simple, the bearing capacity of the soil itself can be fully utilized, and the construction cost is generally low. The disadvantage is that it is cross-constructed with earthwork excavation and earthwork is the main problem.
  Scheme C: it adopts a 1 : 1 grading soil nail wall enclosure scheme; the project site is wasteland, the construction site is very open, and it is not restricted by the red line of the land. According to the principle of optimization, large grading is given priority, the construction process is the simplest, and the surface treatment can be done in time, which can effectively prevent the impact of rainwater on the enclosure.

RETRACTED

The designed schemes are different according to the consideration factors and design preferences. For the same survey results, there are always a variety of feasible schemes for designers or decision makers to choose, as shown in Figure 5.

As shown in Figure 5, the solution in the scientific community is to try to break down the target into layers. It starts from each of its indicators, establishes relationships, and applies decisions based on international engineering experience, so that the problem can be classified into a reasonable range. At the same time, it also makes the decision makers understand the conclusion of this scheme, and the key considerations also appear. The analytic hierarchy process mentioned above is this way of thinking, and many Chinese scholars have applied this method to practical engineering, showing good applicability and feasibility [19, 20].

#### 3.4.2. Principles for Establishing the Indicator System

Considering that there are many factors affecting the selection of the deep foundation pit enclosure scheme and the relationship between them is intricate, in order to be able to systematically, comprehensively, and truly optimize the deep foundation pit enclosure scheme, the index system should be constructed according to the following principles:

The principle of scientificity and comprehensiveness: when constructing the index system, it must be guided by advanced scientific theories, and there must be practical and standardized evaluation methods and evaluation standards [21]. The index system should be able to reasonably and comprehensively reflect the various factors affecting the decision-making scheme, and the concept of the index should be precise and accurate to avoid repetition. By extensively soliciting opinions from experts and relevant technical personnel, the subjective factors of the judges should be minimized.

The principle of combining qualitative analysis and quantitative analysis: the factors are complex and uncertain in the optimal index system of the building envelope. Not all indicators can be accurately quantified, and comprehensive responses need to be combined with qualitative indicators [22, 23].

The principle of combining dynamics and versatility: due to the different types and characteristics of the enclosure structure, the common requirements of enclosure selection should be considered in the design process of the evaluation index system. Therefore, the principle of universality is determined by the nature of the enclosure project itself. At the same time, the surrounding environment of the project is complex and changeable, which will lead to the dynamic characteristics of the evaluation index of the enclosure selection. This requires that the designed index system can reflect it.

### 3.5. Determination of the Comprehensive Index System for Evaluation of Deep Foundation Pit Enclosure Scheme

In order to construct a reasonable evaluation index system of deep foundation pit enclosure scheme, it is necessary to conduct a comprehensive analysis of many factors affecting the deep foundation pit enclosure scheme. Four main index factors were selected from many factors: project cost, construction technology safety, environmental impact, and construction convenience.

#### 3.5.1. Cost of Construction

The cost of construction is an important indicator for the selection of the deep foundation pit enclosure scheme. It is mainly composed of the following aspects: construction cost of enclosure structure, earth excavation cost, construction monitoring and inspection cost, environmental protection cost, etc.

RETRACTED

#### 3.5.2. Safety of Foundation Pit Engineering

Safety is another important indicator for the selection of deep foundation pit enclosure schemes. It mainly includes the following aspects: the stability of the enclosure structure, the development of the engineering experience, the feasibility and reliability of the construction technology, the successful completion of the foundation pit project, and the premise guarantee of construction safety. It is an indispensable indicator in the selection of the foundation pit envelope.

#### 3.5.3. Environmental Impact

Deformation of the enclosure structure and its scope of influence: the deformation of the enclosure structure may cause the surrounding surface subsidence, building damage, etc. Environmental impact caused by construction: this includes mainly the impact of noise, dust, and construction waste during the construction process on the surrounding environment. Feasibility and reliability of environmental protection measures: with the country's emphasis on environmental protection issues and the gradual improvement of the environmental management system, environmental protection has become an important goal in engineering construction.

#### 3.5.4. Difficulty of Construction

For different enclosure schemes, there are often large differences in the degree of difficulty of construction, and this difference will have different degrees of influence on the construction period, quality, and cost of the foundation pit project. The degree of mutual interference between construction procedures is mainly the arrangement of the construction organization. It has a great impact on construction progress and project quality.

In summary, this paper selects the above indicators to construct the index system of the optimal model of the deep foundation pit envelope. The index system constructed in this way can more comprehensively and reasonably optimize the enclosure scheme of the deep foundation pit.

Using *A*_*ij*_ to represent the expert's score for the *i*-th index corresponding to the *j* scheme, then the *n* optimal schemes and the corresponding *m* indexes form an *m*-order *n*-column function evaluation matrix as

(5) $$\begin{array}{c} A=\left[\begin{array}{cccc} a_{11} & a_{12} & ... & a_{1n}\\ a_{21} & a_{22} & ... & a_{2n}\\ ... & ... & ... & ...\\ a_{m1} & a_{m2} & ... & a_{mn} \end{array}\right]={\left(A_{ij}\right)}_{m\times n}. \end{array}$$

Among the indicators of the given impact scheme, there are qualitative indicators and quantitative indicators and the quantitative indicators can directly use the specified values when scoring. The qualitative indicators need to be replaced by reasonable values according to the actual situation and the comparison of the scheme, the indicators are normalized with each other, and the weights are separated for horizontal comparison. Quantitative indicators are relatively objective and effective assessment indicators. The absolute quantity indicators can be production capacity, quality, time, and other quantities. A relative quantity indicator can be any ratio of the same unit quantity.

RETRACTED

The priority needs to determine the corresponding target type; from the engineering indicators, the mathematical model of the corresponding target is given, and then combined with the index values, it constitutes a relative priority matrix.

The evaluation index method is calculated by using the target superiority degree, such as

(6) $$\begin{array}{c} r_{ij}=\left(A_{ij}-A_{j}^{\min}\right)/\left(A_{j}^{\max}-A_{j}^{\min}\right). \end{array}$$

For the index whose score of the scheme index is smaller, the more favorable the project is; the corresponding priority formula is selected as

(7) $$\begin{array}{c} r_{ij}=\left(A_{j}^{\max}-A_{ij}\right)/\left(A_{j}^{\max}-A_{j}^{\min}\right). \end{array}$$

In the formula, *A*_*j*_^min^ and *A*_*j*_^max^ are the lowest and highest scores in the same index.

After the value of each index's superiority is determined, the pros and cons of each scheme are expressed by generalized weighted distance. Weighting means that the weights taken in the adjustment calculation are different due to the different precisions of the measured values. The higher the precision, the greater the weighting. “Weighted” means “multiplied by the weight,” that is, “multiplied by the coefficient.” *D*^+^ is used to express the difference distance between the excellent scheme and the ideal scheme, as shown in the following formula:

(8) $$\begin{array}{c} D^{+}=\mu_{J}^{+}\sqrt{\sum_{i=1}^{m}{\left[W_{i}\left(g_{i}-r_{ij}\right)\right]}^{2}}. \end{array}$$

The difference distance between the optimal solution and the nonideal solution is represented by *D*^−^ as in the following formula:

(9) $$\begin{array}{c} D^{-}=\mu_{J}^{-}\sqrt{\sum_{i=1}^{m}{\left[W_{i}\left(r_{ij}-b_{i}\right)\right]}^{2}}. \end{array}$$

In the formula, *μ*_*J*_^−^ is the membership degree of the corresponding scheme index relative to the optimal scheme index. It can be seen from the formula that if the optimal scheme is taken, that is, the larger each index in a scheme is, the better the objective function which is obtained as

(10) $$\begin{array}{c} F=\min\left|D_{j}^{+2}+D_{j}^{-2}\right|=\mu_{j}^{-2}{\sum_{i=1}^{m}\left[W_{i}\left(r_{ij}-b_{i}\right)\right]}^{2}. \end{array}$$

The objective function is the performance criterion of the system, for example, the lightest weight, the lowest cost, and the most reasonable form of a structure. Let *g*_*i*_=1 and *b*_*i*_=0, *b*_*i*_=0; taking the derivative of the above formula and the solution with the derivative of 0, we obtain as

(11) $$\begin{array}{c} \mu_{j}=1/1+\frac{\sum_{i=1}^{m}{\left[W_{i}\left(1-r_{ij}\right)\right]}^{2}}{\sum_{i=1}^{m}{\left[W_{i},r_{ij}\right]}^{2}}. \end{array}$$

From this, the relative superiority of each scheme can be obtained. According to the principle of maximum membership, the enclosure scheme corresponding to max(*μ*_*j*_) is the optimal scheme. The above process established a satisfactory decision-making mathematical model for the selection of the enclosure scheme.

RETRACTED

### 3.6. Calculation of Evaluation Value of the Selection Index of Enclosure Structure of Deep Foundation Pit

There are many evaluation methods for each index factor in the deep foundation pit enclosure scheme. For example, Analytic Hierarchy Process (AHP) is a systematic and hierarchical analysis method combines qualitative and quantitative analysis. This method quantifies the experience of decision makers and is especially suitable for complex target structures and lack of data. How to choose the appropriate evaluation method according to the actual project will directly affect the evaluation results. In this paper, the satisfaction function is selected as the membership function, namely the evaluation function, based on the careful study of various index factors of deep foundation pit engineering.

By determining the relative superiority matrix of each index to the subsystem and the relative superiority vector of the subsystem to the overall decision, the superiority of each selected bidding scheme to the overall decision is determined. It provides a more objective and fair basis for the final decision-making. The relative superiority degree matrix is a matrix built on the membership degree to determine the superiority degree of each index. In practical applications, the terms that should be used to judge and evaluate the actual situation are used to control the membership range of the method used in the actual situation. The relative favorability matrix should be established in the following format to obtain the following formula:

(12) $$\begin{array}{c} R=\left[\begin{array}{cccc} r_{11} & r_{12} & ... & r_{1m}\\ r_{21} & r_{22} & ... & r_{2m}\\ ... & ... & ... & ...\\ r_{n1} & r_{n2} & ... & r_{nm} \end{array}\right]. \end{array}$$

Membership degree, also known as membership function, is one of the most basic concepts in fuzzy mathematics. For a specific research object with fuzziness, first of all, it is necessary to write a realistic membership function, and then the fuzzy mathematics method can be used for specific quantitative analysis. *m* is the number of membership degrees under the same factor. Assuming that the technical feasibility of the foundation pit enclosure selection scheme is taken as an example, the template of the priority matrix in this paper can be obtained as

(13) $$\begin{array}{c} R=\left[\begin{array}{cccc} r_{11} & r_{12} & ... & r_{17}\\ r_{21} & r_{22} & ... & r_{27}\\ ... & ... & ... & ...\\ r_{51} & r_{52} & ... & r_{57} \end{array}\right]. \end{array}$$

In order to uniformly standardize the evaluation indicators, it is necessary to convert them into standardized values, so that the comparability between different indicators can be achieved. Standardized value calculation is a normal distribution model, and a certain value is a few standard deviations away from the median or the mean. The formula for calculating the normalized value is as follows:

(14) $$\begin{array}{c} L_{i}=\left\{\begin{array}{c} C_{i}/S_{i}\\ S_{i}/C_{i} \end{array}\right). \end{array}$$

In the formula, *C*_*i*_ is the actual calculated value of each index and *S*_*i*_ is the most satisfactory value of this index. The program satisfaction calculation can be calculated in two steps. First, the membership matrix *N* is calculated by multiplying the weight score matrix W by the relative preference matrix *R*, as shown in the following formula:

(15) $$\begin{array}{c} W\cdot R=N. \end{array}$$

Then, multiply the result *N* matrix and the score matrix *P*^*T*^ to get the final satisfaction score *Q*, as shown in the following formula:

(16) $$\begin{array}{c} N\cdot P^{T}=Q. \end{array}$$

The final program selection is determined by the satisfaction score *Q*; the larger the *Q* value, the higher the program satisfaction, and vice versa.

RETRACTED

Because the influence factors of foundation pit enclosure have different influences on foundation treatment, the need for weight distribution is carried out, and the weight value method can be determined by experience or obtained through statistics or expert evaluation. The purpose of setting the weight distribution is to express the degree of satisfaction of the relevant items that need to be checked to the specified requirements with data. It can more intuitively judge the importance of the project to the overall work. In order to get the most accurate results, this paper adopts the expert consultation method and obtains a relatively objective and fair weight value by drawing on the engineering experience of a large number of experts. In this paper, through the survey of 50 experts, the weight distribution opinions of various factors are obtained, as shown in Table 1.

As shown in Table 1, the values corresponding to the five evaluation levels are extremely important, important, relatively important, and should be considered. According to the above opinion parameter table, the weight of each part can be calculated.

### 3.7. Fuzzy Judgment to Determine the Scheme

According to the mentioned model establishment steps, the 3 schemes selected in the preliminary selection are formed into the objective function A. First, 9 indicators are determined by expert evaluation using the method of objective superiority, as shown in Table 2.

As shown in Table 2, it can be seen from the table that each scheme corresponds to the same 9 indicators. By comparing each other with quantitative values, the objective function of 9 indicators is obtained as

(17) $$\begin{array}{c} A={\left[\begin{array}{ccc} 0.7 & ... & 49\\ 0.7 & ... & 74\\ 0.8 & ... & 59 \end{array}\right]}^{T}. \end{array}$$

For the two indexes of the strength condition and stability of the enclosure structure, the larger the index, the more favorable it is to determine its superiority degree, and the smaller the remaining values, the more favorable it is. Because the calculation is complicated, for the convenience of calculation, we edit the corresponding formula in excel, input the target value, and solve the *r*_*ij*_ to obtain the following formula:

(18) $$\begin{array}{c} r_{ij}={\left[\begin{array}{ccc} 0 & ... & 1\\ 0 & ... & 0\\ 1.0 & ... & 0.6 \end{array}\right]}^{T}. \end{array}$$

The weight of each indicator is determined in the fuzzy evaluation method as in the following formula:

(19) $$\begin{array}{c} w={\left[0.0831,0.4355,0.1902,0.1204,0.0403,0.0180,0.0348,0.0123,0.0654\right]}^{T}. \end{array}$$

Since the calculation process is cumbersome, the use of Matlab calculation tools is not widely used in practical engineering and the programming visualization is not high, so the excel table is used in the calculation process, which saves time for similar calculations in the future. Formula (20) can be obtained by the following calculation:

(20) $$\begin{array}{c} \mu_{1}=0.99,\mu_{2}=0.52,\mu_{3}=0.22. \end{array}$$

It can be seen that the upper 4.4 m of the Scheme A corresponding to *μ*_1_ adopts the composite enclosure scheme of 1 : 0.4 grading soil nail wall +15 m slope protection pile +3 prestressed anchor cables as the optimal scheme.

## 4. Economic Subway Stations

At present, the subway has become the first choice for many large and medium-sized cities to alleviate the urban traffic problems. However, subway construction is expensive. According to the statistics of subway projects that have been built in China, the deep foundation pit enclosure of subway stations is shown in Figure 6.

RETRACTED

As shown in Figure 6, the investment is usually 600–800 million yuan per kilometer. It can be seen that the high cost restricts the development of subway construction and there are various factors that affect the comprehensive cost of urban subway projects, such as whether the forecast of passenger flow in the early stage of the subway is accurate, the formulation of subway construction standards, and the rationality of the selection of construction lines.

### 4.1. Constituent Factors and Main Controlling Factors of Subway Construction Cost

In order to fully study the project cost of urban underground excavation subway station, people need to understand the components of the urban subway project cost in detail. Station enclosure costs can generally be divided into initial enclosure and earthwork excavation costs, auxiliary engineering measures costs, construction monitoring costs, transfer channel costs, station decoration costs, and other costs. These items are closely related to the construction process, and the costs affecting the main project cost of the station are shown in Figure 7.

As shown in Figure 7, the design of the subway is usually divided into three stages: general design, preliminary design, and construction design. According to the analysis of subway construction data, the possibility that the overall design stage will affect the project cost is 75%–95%. The possibility of affecting the cost in the preliminary design stage is 35%–75% and the cost in the construction drawing stage is only 20–30%. Therefore, after the feasibility study of the subway project is formulated and implemented, the focus of cost management lies in the design stage.

### 4.2. Suggestions for Reducing Construction Costs

The unique geographical location and geological conditions of the subway station determine the construction methods and procedures used. In order to improve the efficiency and operation effect of the project and achieve the purpose of reducing capital investment, it is necessary to compare and select multiple schemes in combination with the route direction. It also strengthens communication between the cost personnel of the design unit and the subway designers. The construction progress of a subway project is closely related to its cost control, and the two restrict each other. A strict, reasonable, and compact construction schedule is the key to ensuring a reasonable project cost. Of course, measures to ensure construction safety, such as establishing a safety production leading group and improving safety production supervision and inspection agencies, are also powerful guarantees for reducing project costs.

RETRACTED

On the other hand, it is necessary to select correct and reasonable initial enclosure parameters, optimize construction procedures, and reduce auxiliary works. Subway projects should be smoothly dismantled, surveyed, and scientifically planned. The subway route should be selected along the main roads of the city as much as possible, and the amount of dismantling work should be greatly reduced, and the subway project during the construction process should be reduced.

## 5. Experiment and Comparison and Selection of the Deep Foundation Pit Envelope Structure Scheme

### 5.1. Investigation and Metro Development

Since the implementation of the policy of reform and opening up, China's economy has developed rapidly, the process of urbanization has been accelerated, the scale of cities has gradually increased, and the number of urban population has increased dramatically. The built urban roads have been unable to adapt to the surge in the flow of people and vehicles, and it is difficult to meet the travel of citizens, especially in big cities, where traffic congestion and disorder are very serious, as shown in Figure 8.

As shown in Figure 8, in view of the increasing shortage of urban land resources, it is suitable for the actual situation of Chinese cities and the transportation structure system combining urban rail, interchange, and expressway in large and medium-sized cities. Therefore, in the past ten years, subway construction has ushered in an unprecedented period of development. Dozens of cities have successively carried out subway construction and put into operation, and they have done a great job.

The purpose of the experiment in this paper is to monitor the structural deformation of the foundation pit and the surrounding buildings. It timely understands the soil layer change information during the construction process, the envelope structure deformation under various working conditions, and the impact on the surrounding buildings and the environment. It realizes the information construction management to ensure the safety and reliability of the foundation pit project and the normal use of the buildings and underground pipelines around the foundation pit. In this paper, the stability, security, and economy of the three schemes are compared and analyzed.

### 5.2. Monitoring of Three Deep Foundation Pit Enclosure Structures

This paper specially invited 5 experts to score the 3 schemes, as shown in Tables 3–5.

RETRACTED

As shown in Tables 3–5, from the experts' scores for the three schemes, each expert tends to scheme A, and among the three schemes, the scores obtained are also very high. In Scheme A, the lowest score given by 5 experts is 8.0 and the highest score is 9.3. In other schemes, the highest scores are 7.9 and 7.5 points. It is conceivable that Scheme A is the best scheme. However, sometimes the accuracy of this scoring method is not high, and it may also have personal subjective awareness. Therefore, in order to verify the feasibility of the scheme, the excavation project was monitored in this experiment.

The excavation process of the foundation pit will inevitably have a great impact on the underground pipeline. This foundation pit project has monitored the surrounding surface and the vertical displacement curve of the surface around the foundation pit is shown in Figure 9.

As shown in Figure 9, when the foundation pit is excavated, the inner side of the foundation pit is unloaded, causing the active earth pressure above the excavation surface to increase, resulting in a large vertical displacement of the surrounding surface. When the prestressed anchor cable is tensioned and locked, the increase of active earth pressure on the envelope structure is limited. The vertical displacement of the ground around the foundation pit of Scheme A gradually tends to be stable.

In three calculation modes, the deep foundation pit Lizheng software gives the settlement and displacement data of the ground surface at a certain distance from the edge of the foundation pit. The monitoring point of surface settlement and displacement on the north side of the foundation pit is arranged on the outside of the rear row of piles, about 4.8 m away from the pit edge, as shown in Figure 10.

As shown in Figure 10, in the calculation results of the deep foundation pit design, the distance from the edge of the foundation pit is 4.8 m and the maximum settlement in the three modes is: 60 mm for the parabolic method, 63 mm for the triangle method, and 68 mm for the exponential method. The measured settlement of the ground surface is much smaller than the above values, the calculation of deep foundation pit is relatively conservative, and the safety is relatively high. According to the data obtained by monitoring, it tests the rationality of the design scheme. It provides accurate feedback for timely improvement of design parameters and revision of construction processes. It ensures the safe operation of foundation pit engineering, and it enables subsequent structural engineering to achieve good engineering results.

## 6. Conclusion

In today's era, the rapid progress of computer technology and the rapid development of on-site construction technology have also promoted the development of deep foundation pit enclosures in subway stations. With the increasing traffic pressure, more and more people are willing to take the subway to travel, which not only saves people's time but also saves a lot of money. The construction and operation of subway can promote the development of industry, transportation, real estate, and other related industries, stimulate employment, promote the appreciation of land along the way, and expand the space for urban development. It has obvious external economy. However, this also makes the construction of the deep foundation pit of the subway station more difficult. Therefore, this paper compares and selects the construction scheme of the deep foundation pit of the subway station, and analyzes the economy. Using fuzzy logic, this paper proposes a fuzzy comprehensive evaluation method to evaluate the scheme. This paper proposes 3 different schemes, and finally it concludes that Scheme A is the most feasible scheme. It is not only safe but also very economical. In the experimental part, the scheme is tested again, and it is found that the stability of Scheme A is also very strong. Therefore, after comprehensive consideration, the scheme selected in this paper is Scheme A. In a word, the comparison and selection of the deep foundation pit envelope structure scheme of the subway station have a great influence on the subway construction.

RETRACTED

## Figures and Tables

**Figure 1:** Schematic diagram of deep foundation pit enclosure.

**Figure 2:** Simple enclosure of foundation pit. (a) Earthbag or block stone stacking enclosure. (b) Short pile enclosure.

**Figure 3:** Enclosure form of soil nailing wall.

**Figure 4:** Internally braced envelope structure.

**Figure 5:** Factors that should be considered in the scenario.

**Figure 6:** Deep foundation pit enclosure of the subway station.

**Figure 7:** Costs affecting the cost of main projects of the station.

**Figure 8:** Growth trend of the number of people who choose to travel by subway from 2015 to 2020.

**Figure 9:** The vertical displacement of the ground around the foundation pit under the three schemes.

**Figure 10:** Monitoring data of surface subsidence.

**Table 1:** 50 experts' opinions on the weight distribution of each factor.

Target	Extremely important	Important	More important	Should be considered
Strength condition of support structure	43	7	0	0
Stability	38	10	2	0
Maximum deformation	27	13	10	0
Engineering impact	25	11	14	0
Construction impact	20	21	8	1
Possibility of secondary disasters	16	18	15	1
Difficulty in construction	18	20	10	2
Mutual interference	15	31	1	3
Construction period	10	21	15	4

RETRACTED

**Table 2:** The value of the merit of each indicator.

Target	Scenario A	Scenario B	Scenario C
Strength condition of support structure	0.8	0.7	0.7
Stability	1.5	1.4	1.2
Maximum deformation	24	27	27
Engineering impact	0.6	0.8	0.84
Construction impact	0.7	0.9	0.84
Possibility of secondary disasters	0.84	0.7	0.7
Difficulty in construction	0.8	0.84	0.7
Mutual interference	0.7	0.84	0.84
Construction period	59	74	49

**Table 3:** 5 experts' rating of Scheme A.

Expert	Safety	Technically feasible	Convenient construction
Expert 1	8.9	8.8	9.0
Expert 2	8.6	8.4	8.1
Expert 3	9.3	8.6	8.5
Expert 4	9.0	8.0	8.7
Expert 5	9.1	8.9	8.2

**Table 4:** 5 experts' ratings for Scheme B.

Expert	Safety	Technically feasible	Convenient construction
Expert 1	7.9	7.3	6.4
Expert 2	7.4	7.2	6.6
Expert 3	7.3	6.8	6.3
Expert 4	7.6	6.9	6.7
Expert 5	7.8	6.5	6.2

**Table 5:** 5 experts' ratings for Scheme C.

Expert	Safety	Technically feasible	Convenient construction
Expert 1	6.5	6.2	5.8
Expert 2	6.9	6.1	5.3
Expert 3	6.6	7.5	5.5
Expert 4	6.2	7.2	5.4
Expert 5	6.3	7.0	5.6

## Data Availability

No data were used to support this study.
